# Mechanisms of Tolerance and High Degradation Capacity of the Herbicide Mesotrione by *Escherichia coli* Strain DH5-α

**DOI:** 10.1371/journal.pone.0099960

**Published:** 2014-06-12

**Authors:** Luiz R. Olchanheski, Manuella N. Dourado, Flávio L. Beltrame, Acácio A. F. Zielinski, Ivo M. Demiate, Sônia A. V. Pileggi, Ricardo A. Azevedo, Michael J. Sadowsky, Marcos Pileggi

**Affiliations:** 1 Universidade Estadual de Ponta Grossa, UEPG, Departamento de Biologia Estrutural, Molecular e Genética, Ponta Grossa, PR, Brazil; 2 Escola Superior de Agricultura Luiz de Queiroz, ESALQ, Universidade de São Paulo, USP, Piracicaba, SP, Brazil; 3 Universidade Estadual de Ponta Grossa, UEPG, Departamento de Ciências Farmacêuticas, Ponta Grossa, PR, Brazil; 4 Programa de Pós-Graduação em Engenharia de Alimentos, Universidade Federal do Paraná, Curitiba, PR, Brazil; 5 Universidade Estadual de Ponta Grossa, UEPG, Departamento de Engenharia de Alimentos, Ponta Grossa, PR, Brazil; 6 Department of Soil, Water, and Climate, and BioTechnology Institute, University of Minnesota, St. Paul, Minnesota, United States of America; University Paris South, France

## Abstract

The intensive use of agrochemicals has played an important role in increasing agricultural production. One of the impacts of agrochemical use has been changes in population structure of soil microbiota. The aim of this work was to analyze the adaptive strategies that bacteria use to overcome oxidative stress caused by mesotrione, which inhibits 4-hydroxyphenylpyruvate dioxygenase. We also examined antioxidative stress systems, saturation changes of lipid membranes, and the capacity of bacteria to degrade mesotrione. *Escherichia coli* DH5-á was chosen as a non-environmental strain, which is already a model bacterium for studying metabolism and adaptation. The results showed that this bacterium was able to tolerate high doses of the herbicide (10× field rate), and completely degraded mesotrione after 3 h of exposure, as determined by a High Performance Liquid Chromatography. Growth rates in the presence of mesotrione were lower than in the control, prior to the period of degradation, showing toxic effects of this herbicide on bacterial cells. Changes in the saturation of the membrane lipids reduced the damage caused by reactive oxygen species and possibly hindered the entry of xenobiotics in the cell, while activating glutathione-S-transferase enzyme in the antioxidant system and in the metabolizing process of the herbicide. Considering that *E. coli* DH5-α is a non-environmental strain and it had no previous contact with mesotrione, the defense system found in this strain could be considered non-specific. This bacterium system response may be a general adaptation mechanism by which bacterial strains resist to damage from the presence of herbicides in agricultural soils.

## Introduction

In recent years, there has been a high demand for increasing agricultural productivity and the arable land area, accompanied by the large scale use and discovery of new pesticides and fertilizers [1]–[3]. It was estimated that approximately 2.27 million tons of agrochemicals were released into the environment in 2001, 35% of which were herbicides [4]. Despite the fact that the use of pesticides in agriculture has had a positive impact on crop productivity, concerns have been expressed about the adverse effects of these chemicals [5], since only 0.1% of them reach their specific targets. For this reason, there is a large quantity of herbicide residues remaining in the environment, which can be metabolized by microbiota [6]–[8].

Herbicide application has brought damage to the soil microbiota, and may have affected the dynamics of biogeochemical cycles and soil fertility. The herbicide napropamide, for example, has been identified as harmful to soil functionality, based on the structural and functional diversity of the soil bacterial community [9]. Other studies have demonstrated the inhibition of nitrification and changes in ammonia oxidation in soils by the herbicide simazine [10]. As regard to the triketone herbicides mesotrione and sulcotrione, their toxicity level was considered equal to or higher than atrazine in studies with model organisms, such as *Tetrahymena pyriformis* and *Vibrio fischeri* [11].

Bioremediation has been the main strategy used to eliminate xenobiotics, mainly herbicides, from the environment, and this subject has been the focus of many biotechnological studies [12]–[13]. Degradation processes mediated by microorganisms in large part influence the persistence of herbicides in the soil [14].

Reactive oxygen species (ROS), apart from being part of normal aerobic metabolism [15], may increase in concentration as a result of exposure to toxic substances, as for example, when bacteria come into contact with herbicides [16]. An increase in the rate of hydrogen peroxide (H_2_O_2_), and superoxide (O^2−^) and hydroxyl (OH^•^) radicals production can cause damage to DNA, RNA, proteins and lipids [17]–[18]. An efficient antioxidant enzyme system is the primary line of defense for the elimination of excess ROS, such as the action of catalase, superoxide dismutases, peroxidases and glutathione reductase [15]. Glutathione-s-transferase (GST), as well as participating in the system of redox homeostasis and response to ROS [19]–[20], catalyzes the conjugation of glutathione with herbicides, and it can operate to degrade some herbicides, also being responsible for resistance to antibiotics [21].

Mesotrione (Fig. 1) is the active ingredient of the herbicide Callisto; it has a selective action and is recommended for the systematic control of weeds in maize cultivation, both in pre and post-planting applications. This molecule is derived from a phytotoxin that is produced by the plant *Callistemon citrinus*, and it inhibits the enzyme 4-hydroxyphenylpyruvate dioxygenase (HPPD), acting in the conversion of tyrosine to plastoquinone and α-tocopherol. The inhibition of plastoquinone leads to an interruption of the carotenoid synthesis pathway, causing the death of leaf tissues [22]–[23]. In mesotrione-tolerant plants, the metabolism of the herbicide is mainly carried out by the enzyme P450 [24]–[25]. A P450-like, synthesized by *cysj* gene, was reported in reducing paraquat herbicide in bacteria [29]. But glutathione S-transferase (GST) is also involved in the detoxification of herbicides of the triketone family [26], and in the metabolism of herbicides on microorganisms [27]–[28].

**Figure 1:** Molecular structure of mesotrione.

The degradation products of mesotrione by a *Bacillus* sp. strain were found to be 4-methylsulfonyl-2-nitrobenzoic acid (MNBA) and 2-amino-4-methylsulfonylbenzoic acid (AMBA) [30]-[31]. AMBA has been characterized as being more toxic than the original molecule [11]. Studies with *Pantoea ananatis* have demonstrated the degradation of mesotrione by a different route, with metabolic products probably less toxic than the original molecule (C_13_H_10_NO_7_S, C_11_H_13_O_8_S and C_11_H_11_O_7_S) [32]. The presence of MNBA and AMBA was reported in soils treated with high concentrations of mesotrione [33].

Strains of *E. coli* are currently used to determine the toxic effects of xenobiotics [34]. This model organism [35] has been widely used in recombinant DNA technology [36]. So far, no studies of degradation capacity have been carried out without a prior modification of *E. coli* strains.

Given the toxic effect of herbicides on bacteria, we aimed to assess whether a laboratory, non-environmental strain *E. coli* (DH5-α) possessed any mechanism of adaptation to mesotrione, even with no previous contact with this herbicide.

## Materials and Methods

### Bacterial strain

The *Escherichia coli* strain DH5-α [(genotype: F^−^φ80dlacZΔM15 Δ(lacZYA-argF) U169 deoR, recA1 endA1 hsdR17 (r_k_^−^ m_k_^+^) phoA supE44λ^−^ thi-1 gyrA96 relA1)] was used to evaluate the degradation of mesotrione herbicide.

### Herbicides

Mesotrione (99% purity) was provided by Syngenta Crop Protection, Greensboro, NC (USA). For HPLC (High Performance Liquid Chromatography) experiments, the analytical standard Pestanal (99% pure) (Sigma-Aldrich) was used.

### Evaluation of herbicide degradation by HPLC

In order to determine the mesotrione degrading ability of *E. coli*, the strain was grown in 100 mL of LB (Luria Broth: 10 g L^−1^ tryptone; 5 g L^−1^ yeast extract; 10 g L^−1^ NaCl) in 250 mL flasks, and incubated at 37°C, at 200 rpm. The cells were collected after 10 h and centrifuged at 8,000×*g* for 10 min. at 4°C. The pellet was washed twice with PBS (pH 6.8, phosphate buffered saline: 8 g L^−1^ NaCl; 0.2 g L^−1^ KCl; 1.44 g L^−1^ Na_2_HPO_4_; 0.24 g L^−1^ KH_2_PO_4_), and cells were re-suspended in 10 mL of MMM (Mineral Medium with Mesotrione: 3 g L^−1^ NaNO_3_; 0.5 g L^−1^ MgSO_4_; 0.5 g L^−1^ KCl; 0.01 g L^−1^ FeSO_4_; 0.04 g L^−1^ CaCl_2_; 0.001 g L^−1^ MnSO_4_; 0.4 g L^−1^ glucose, 0.04 mM mesotrione; 10 mM potassium phosphate buffer, pH 7.0;). This corresponded to 1×, or normal field levels according to manufacturer's instruction. Cells were placed in mineral medium without carbon source (-CM), with five repetitions, and incubated at 37°C, at 200 rpm. For analysis of herbicide adsorption by bacteria, cells were boiled prior to being added to the treatments already described. As a negative control, a flask with MMM was incubated, in the same conditions, without *E. coli* DH5-α. Aliquots (1 mL) were collected from the culture medium every hour of incubation (from 0 to 12 h) and centrifuged at 13,000 *g* for 5 min. The supernatant (0.9 mL) was frozen for further HPLC analysis.

Samples were filtered with 0.22 µm syringe filters and HPLC analysis was performed using a Waters Alliance e2695 and a photodiode detector (Waters 2998 PDA), adjusted at a wavelength of 254 nm. An Eclipse XDB-C18 column was used, with dimensions of 4.6 mm×150, at 3.5 µm for separation, at 20°C. The gradient of the mobile phase started with 70% water (0.1% phosphoric acid) (A): 30% acetonitrile (B); 30% B for 3 min.; 55% B for 15 min.; 100% B for 17 min.; 100% B for 18 min.; 30% B for 19 min. and 30% B for 29 min., for conditioning the column to a new injection). The flow rate was 1 mL min^−1^. The injection volume of the samples was 50 µL. The HPLC method was developed, validated and applied to analysis of mesotrione degradation rate.

### Cell viability

Bacteria were grown for 10 h at 37°C in 1.2 L of LB. Cells were centrifuged at 8,000×*g* for 10 min., washed twice with PBS, and divided into vials containing 50 mL of MM (control), MMM (mineral medium with mesotrione), -C (MM without carbon source) and -CM (MMM with mesotrione as sole carbon source), with three repetitions. The flasks were incubated at 37°C (at 200 rpm), and 100 mL aliquots were withdrawn after 30 min., 3 h and 6 h of incubation. Samples were diluted to 10^−8^, plated on LB medium and incubated at 37°C. After 12 h, the colony forming units (CFU) counting was determined.

### Lipid peroxidation

Lipid peroxidation was determined by the levels of malondialdehyde (MDA) (substances reactive to thiobarbituric acid) [37]. The concentrations of MDA were monitored at 535 and 600 nm, and their concentrations were calculated using an extinction coefficient of 155 mM cm^−1^.

### Protein extraction for analysis of oxidative stress

Bacteria were grown for 10 h at 37°C (at 200 rpm) in 3.6 L of LB, to get enough cells for the following steps of protein extraction. The cells were centrifuged at 8,000×*g* for 10 min., washed twice with PBS, and divided into vials with 50 mL of MM (control), MMM, -C (MM without carbon source), and -CM (MMM with mesotrione as sole carbon source), with three replications. All the flasks were incubated at 37°C, and extractions were performed at 30 min., 3 h, and 6 h.

For enzyme extraction, the cultures were centrifuged at 8,000×*g* for 10 min., and the pellet was macerated with liquid nitrogen, and homogenized (10∶1 w/v) in 100 mM potassium phosphate buffer (pH 7.5), containing 1 mM ethylenediaminetetraacetic acid (EDTA), 3 mM DL-dithiothreitol and 5% (w/v) polyvinylpolypyrrolidone [38], always kept at 4°C. The homogenate was centrifuged at 10,000×*g* for 30 min., and the supernatant was divided into aliquots, and frozen at −80°C for subsequent enzyme analysis. The protein concentration was determined by the Bradford method [39], using BSA as standard.

### Protein analysis by polyacrylamide gel electrophoresis (PAGE)

Electrophoresis was performed in gels containing 12% polyacrylamide with 4% stacking gel. For SOD-PAGE, SDS was eliminated. A current of 15 mA gel^−1^ was applied for 3 h (SOD activity gel) at 4°C or 2 h (protein profile gel) at room temperature. Equal amounts of protein (20 µg) were applied to the gels. For SDS-PAGE, the gel was washed with distilled water, and incubated overnight in 0.05% Coomassie blue R-250 solution, at a ratio of 40∶7∶53 of methanol:acetic acid:water (v/v/v), and decolorized by successive washings with a solution, at a ratio of 40∶7∶53 of methanol:acetic acid:water (v/v/v) [40].

The SOD-PAGE activity was performed according to Beauchamp and Fridovich [41] and modified by Medici et al. [42], in which the gels were washed in distilled water, and incubated in the dark for 30 min. in 50 mM potassium phosphate buffer (pH 7.8), containing 1 mM EDTA, 0.005 mM riboflavin, 0.1 mM nitroblue tetrazolium, and 0.3% N,N,Ń,Ń-tetramethylethylenediamine. To control the reaction, a unit of bovine liver SOD (Sigma) was used. The gels were exposed to white light and immersed in water until the development of the SOD bands.

### Catalase (CAT) activity

CAT activity was determined according to Kraus et al. [43] in a solution containing 1 mL of potassium phosphate buffer 100 mM (pH 7.5) and 2.5 µL H_2_O_2_ (30% solution), and quantified in a spectrophotometer at 25°C. The reaction was initiated with the addition of 25 µL of protein extract, and the activity was determined by following the decomposition of H_2_O_2_ at 240 nm for 1 min.

### GST activity

GST activity was measured in a solution containing 900 µL of potassium phosphate buffer 100 mM (pH 6.8), adding 25 µL of 1-chloro-2,4-dinitrobenzene (CDNB) 40 mM and 50 µL of reduced glutathione (GSH) 0.1 M, and incubated at 30°C [44]. The reaction was initiated with the addition of 25 µL of protein extract, and was monitored for 2 min. at 340 nm.

### Analysis of lipids saturation

Bacterial strain was grown in 800 mL of LB and incubated at 37°C, at 200 rpm. After 12 h, the samples were centrifuged at 8,000×*g* for 5 min. at 4°C. The pellet was washed twice with PBS and divided into vials containing 50 mL with LB and LB plus 0.04 mM mesotrione, in triplicate, and the cultures were incubated at 37°C, at 200 rpm. After 12 h, lipid extraction was performed, as described by Bligh and Dyer [45], with modifications. The membrane lipids were analyzed by FTIR (Fourier Transform Infrared Spectroscopy) with transmittance at wavelengths from 400 to 4,000 cm^−1^.

### Experimental design and statistical analysis

To assess the saturation of lipids, the baseline of spectrums were corrected, and then processed by PCA (Principal Component Analyzes) implemented in the Pirouette v. 4.0 software (Infometrix, Bothell, WA, USA). PCA was applied to separate the samples according to their FTIR spectra (1,400 to 3,200 cm-1). Therefore, the results obtained for each wavelength were plotted as columns and the samples as rows. Mean-Center was used as pre-treatment of the results.

Statistical analysis were conducted with three repetitions of each treatment for cell viability, MDA, GST and CAT experiments, which were performed in a completely random design. The significance of the observed differences was verified using a one-way analysis of variance (*P*<0.05). Analysis were made using R software version 3.0.1.

## Results and Discussion

### Mesotrione degrading capacity by *E. coli* DH5-α

*E. coli* is considered a model bacterium for study the physiology of prokaryotes [35]. Studies have been using the *E. coli* DH5-α strain as a recipient of genetic material, and it is one of the strains most frequently used as a tool in recombinant DNA technology [36], [46]–[47]. Thus, we considered this strain as a laboratory, non-environmental bacterium, with no prior contact with herbicides.

The *in vitro* evaluation of the toxic effects of herbicides revealed a negative effect on the growth of strains of *E. coli*, particularly at higher doses [34], and also served as a model for the identification of genes and enzymatic activities involved in the antioxidant system in general [48]–[50]. Until this date, there are no studies involving herbicides degrading ability by non-environmental strains as *E. coli* DH5-α.

According to Batisson et al. [51], in high concentrations, mesotrione can alter the microbial community, selecting tolerant or degrading strains. *Bacillus* sp. 3B6 [52] and *P. ananatis* CCT 7673 [32] have been described as capable to degrade mesotrione in 24 h and 18 h, respectively. Similarly, *E. coli* DH5-α biotransformed mesotrione, and after 3 h of exposure to MMM, no compound was detected in the analyzed samples, and 76% in –CM (Fig. 2). The boiled cells test showed that mesotrione was not lost from the culture medium by cell adsorption. In contrast, *P. ananatis* CCT 7673 showed no ability to metabolize the herbicide without the presence of carbon [32].

**Figure 2:** Degradation kinetics of mesotrione mediated by *E. coli* DH5-α. MMM (mineral medium with mesotrione), -CM (mineral medium without carbon, with mesotrione), negative control (MMM without *E. coli* DH5-α) and boiled cells.

In studies of mesotrione degradation in soil, it was observed that the highest rate of degradation of Callisto occurred with the application of 10× and 100× [33]. *P. ananatis* CCT 7673 (a strain isolated from water) was able to completely metabolize the herbicide mesotrione, but could not grow when in contact with the herbicide at high doses [32]. In our studies, *E. coli* DH5-α was able to tolerate and degrade the herbicide in 10× and in a shorter incubation time. The tolerance exhibited by this bacterium to the herbicide may be explained by its rapid metabolism, since the degradation process takes place as soon as the strain is exposed to the xenobiotic, reducing the time of exposure of the bacterium to the chemical.

Studies of mesotrione degradation reported difficulty in finding specific genes for the degradation of this herbicide [23], [43]. According to Pileggi et al. [32], the strains *E. coli* DH5-α, TOP 10, and K-12 have the ability to metabolize mesotrione. Considering that they are related to strains developed in the laboratory, with no prior contact with the herbicide, this fact may indicate low selective pressure for specific genes to degrade mesotrione.

### Characterization of mesotrione herbicide as a stress agent

In order to determine if mesotrione damaged cells of *E. coli* DH5-α, its cellular viability was assessed under the same growth conditions as for protein extraction (Fig. 3). The data obtained revealed that the herbicide mesotrione was not detected after 3 h exposure (Fig. 2) and that the metabolic process was shown to initiate in the first hour of growth; therefore, the *E. coli* DH5-α strain was probably in contact with the whole herbicide for at least the initial growing of 30 min. During this period, a decrease in cell viability was observed in the treatments with the herbicide (MMM and -CM), compared with the controls (MM and -C) (Fig. 3), indicating a toxic effect of the herbicide on the *E. coli* DH5-α. During the periods of 3 h and 6 h, similar viability rates were verified for all treatments, which is probably due to the capacity of the nutritional support from MM provided to the bacterial cells.

**Figure 3:** Cellular viability of *E. coli* DH5-α in MM and in the MMM, -C and –CM treatments, during the periods of 30 min., 3 h and 6 h. LSD = 0.13 for all pairwise comparison.

Botelho et al. [34] analyzed many widely used commercial formulations of herbicides, and only paraquat decreased the growth of the *E. coli* ATCC 25922 strain. In the present study, field doses (1×) of mesotrione, which is considered less toxic than the commercial herbicide [22], decreased the viability of *E. coli* DH5-α within 30 min. in treatments with the herbicide (MM and -CM) (Fig. 3).

Balagué et al. [53] used doses of 2 mM, 1 mM, 0.1 mM and 0.01 mM of the herbicide 2,4-D in spectrophotometer analysis, and verified growing inhibition of *E. coli* HB101 only at 2 mM, whilst in the present study, the growth capacity, analyzed by cellular viability, showed significant differences in *E. coli* DH5-α between control and mesotrione treatments in 30 min. evaluation (Fig. 3).

The malondialdehyde (MDA) rate has been used as an indicator of lipid peroxidation in other studies involving oxidative stress, such as that reported by Lima and Abdalla [54]. In the present study, *E. coli* DH5-α exhibited lower membrane damage, in the -CM treatment, within 30 min., while mesotrione still remained in the culture medium, (Fig. 4). Although cell viability was affected by the presence of mesotrione (Fig. 3), in the three analyzed times, the rates of MDA measured did not show an increased lipid peroxidation, in the -CM treatment. Nevertheless, in the MMM treatments, during all the periods analyzed, a statistically significant increase in MDA was observed, suggesting an imbalance in ROS production/ROS homeostasis, and consequently a toxic effect of the extra ROS was produced.

**Figure 4:** MDA levels in *E. coli* DH5-α in MM, and in the MMM, -C and -CM treatments, during periods of 30 min., 3 h and 6 h, respectively. LSD = 0.18 for all pairwise comparison.

### Influence of mesotrione on the level of lipids

Infrared spectrogram analysis showed changes in the structure of the membrane lipids of *E. coli* DH5-α in the presence of the herbicide mesotrione (Fig. 5). According to Böger et al. [55], an increase in the proportion of unsaturated fatty acids in bacterial cell membranes, makes them more susceptible to attack by ROS, and induces to higher rates of MDA production. These changes in membrane lipids occur from chloroacetanilide herbicides. A study by Balangué et al. [53] with *E. coli* HB101 strain demonstrated that the toxicity of 2,4-D could reduce the fluidity of bacterial membrane, and consequently alter MDA results, as a system-wide response against ROS. Sánchez et al. [56] also reported similar findings, where the strain *Klebsiella planticola* DSZ, when in contact with ethanol or the herbicide simazine, exhibited a decrease in the saturation of membrane lipids, altering the rate of selective permeability, possibly as a defense system.

**Figure 5:** Analysis of lipids of *E. coli* DH5-α using FTIR and principal component analysis. Points M2 and M5: control without mesotrione (LB), in duplicate. Points M1, M3 and M4: treatment with mesotrione (LB+0.04 mM mesotrione) in triplicate. Point B2: negative control, *Bacillus* sp. in the absence of mesotrione.

In the present study, such a change in the composition of the membrane lipids of *E. coli* DH5-α may explain the lower rate of MDA in the treatments without the presence of carbon and with mesotrione (Fig. 4), as shown by data from cell viability (Fig. 3), in which the presence of mesotrione caused damage to bacteria in a time of 30 min. Apart from defense against ROS, the change in selective permeability may have prevented the entrance of mesotrione, with increased saturation of membrane lipids, characterizing a defense system against xenobiotics.

### Involvement of antioxidant enzymes in the defense and degradation of mesotrione

By superoxide dismutase gel analysis, up to 6 distinct isoenzymes (Fig. 6, lane 3) were observed among the treatments used (Fig. 6). These isoenzymes were not necessarily present in all treatments, but the majority of the SOD activity detected could be accounted to SOD I and SOD IV isoenzymes. A larger number of bands were always observed when *E. coli* DH5-α was in MM (Fig. 6, lane 3) and MMM (Fig. 6, lane 6), at 6 h of exposure/growth. The higher SOD activity observed, under such conditions, and based on the higher intensity of the SOD bands, could be attributed to the increased number of visible SOD bands, and also to the higher activity of SOD I and SOD IV isoenzymes, which together clearly accounted for the majority of the SOD activity in *E. coli* DH5-α. Yet, it is likely that this difference on band intensity was due to the incubation time of *E. coli* DH5-α, and consequently occurred an increase of superoxide radical production. As shown in the treatment with carbon (MM and MMM), as longer the growing time, the higher was SOD activity. However, this was not observed in the treatment without carbon (-CM). Ongoing research is classifying the distinct SOD isoenzymes, as proposed by Azevedo et al. [57], detecting which shall be important in future studies, since they may be located in distinct cell compartments, and consequently allow to link an increase in superoxide in a specific organelle to an specific increase of one or another particular SOD isoenzyme.

**Figure 6:** Non-denaturing-PAGE for SOD activity. Patterns presented by *E. coli* DH5-α in MM (lines 1, 2 and 3) and in the MMM (lines 4, 5 and 6), -C (lines 7, 8 and 9), and -CM (lines 10, 11 and 12) treatments, at periods of 30 min., 3 h and 6 h, respectively.

An increase in CAT activity was observed, depending on the exposure time in the culture media with the presence of carbon (MMM and MM) (Fig. 7), which was probably due to the adaptation and growth of the strain in the mineral medium. However, there were no differences in relation to the presence of mesotrione. In strains of *E. coli*, depending on the growth phase, different isoforms can act, which have regulatory pathways that are activated independently [58]. This may have influenced the CAT activity response and also the potential participation of other peroxidases in the stress response.

**Figure 7:** CAT activity in *E. coli* DH5-α in MM, and in the MMM, -C and -CM treatments, at periods of 30 min., 3 h and 6 h, respectively. LSD = 1.17 for all pairwise comparison.

In the culture media without carbon (-C and -CM), despite showing a significantly lower total CAT enzymatic activity, in comparison with the media with carbon, the activity of CAT was higher in the media with mesotrione, except in 3 h exposure period (Fig. 7). In the period of 30 min., during which the complete degradation of the herbicide had not yet occurred, and mesotrione appeared as the only carbon source, the amount of hydrogen peroxide may have increased in response to the xenobiotic itself, stimulating CAT activity, which is notable when compared to the control without carbon source (-C).

In relation to *E. coli* DH5-α, GST activity was higher in the 30 min. exposure treatments in the presence of mesotrione, compared to medium without the herbicide. However, in the 3 h period, no differences occurred in the activities of GST (Fig. 8). There are reports about metabolization of triketone herbicides (such as mesotrione) by influence of cytochrome P450 in plants [24]–[25]. According to Barrett [24], P450 is essential for the biodegradation of at least six families of herbicides used in maize culture. Furthermore, both the P450 as GST are involved in cellular defense and detoxification of these herbicides in maize and rice [26].

**Figure 8:** GST activity of *E. coli* DH5-α in MM, and in the MMM, -C, and -CM treatments, at periods of 30 min. 3 h and 6 h, respectively. LSD = 0.000398 for all pairwise comparison.

The involvement of the cytochrome P450 enzyme system in degradation of atrazine and herbicides EPTC (*S*-Ethyl Dipropylthiocarbamate) was observed in bacteria [59]–[60], but at a very slow rate [61]. A P450 like enzyme,synthesized by the *cysj* gene, is involved only in the reduction pathway of paraquat in *E. coli*, not in the degradation[29], thereby changing the mode of action of this herbicide [62].

On the other hand, GST enzymes have been characterized in plants and microorganisms, as mechanisms aiding the metabolism of herbicides and other toxic products, catalyzing the conjugation of glutathione with the herbicide and marking the compound to be degraded [27]–[28]. However, there is a great diversity in this enzyme, with various functions still unknown [21], [63]–[64].

*E. coli* DH5-α strain exhibited the capacity to transform 100% of mesotrione in only 3 h of exposure (Fig. 2). Taking into account the GST activity during the period in which the degradation rate is high (30 min.), and any other enzyme related to mesotrione degradation was reported in bacteria, there is a possibility that this enzyme is involved in the process of degradation of the herbicide, because during the period of 3 h, when the herbicide was completely degraded, the GST activity decreased (Fig. 8). Besides, acting on the first transformation of the herbicide, the GST enzyme may also be involved in the elimination of ROS and in the adaptation of the strain to the culture medium [65]–[67]. The evaluation of CAT (Fig. 7) and SOD enzymes (Fig. 6) provides evidence that these enzymes showed no specific changes in activity in response to the herbicide in *E. coli* DH5-α. Such a response may vary, as shown by Martins et al. [13], who also failed to see specific changes in SOD activity that could be attributed to the herbicides (acetochlor and metolachor), but observed specific changes in CAT activity by the same bacterial isolates and to the same herbicides. Thus, it appears that GST may be acting directly in defense against ROS and in the degradation of mesotrione by *E coli* DH5-α.

## Conclusions

This is the first report showing that *Escherichia coli* DH5-α, which is considered a non environmental strain, was able to degrade mesotrione without previous exposure to the herbicide The process of degradation took only 3 h, being the lowest degradation time reported until now. Previous articles tried to discover a gene responsible for mesotrione degradation, without success. In this manuscript, we describe the involvement of GST in herbicide degradation, as part of a more complex response system to mesotrione. Nevertheless, it cannot be ruled out that other systems may also be involved cooperatively or independently, such as other peroxidases.

Mesotrione was identified as an oxidative stress agent by the involvement of GST in herbicide degradation, changes in membrane lipids saturation, preventing membrane cell peroxidation, and differences in cellular viability. In this case, MDA did not indicate the occurrence of cellular damage by oxidative stress, but its reduction was related to changes on lipid structure in response to the herbicide. To our knowledge, this manuscript is the first report on the characterization of mesotrione as an oxidative stress agent in bacteria. Nevertheless, we described *Escherichia coli* DH5-α as a tolerant strain and capable of growing in the presence of the herbicide at concentrations normally used in the environment by agricultural management, even without previous contact with the herbicide. We consider that *E. coli* strains can manage to adapt to the presence of new synthesized toxic molecules in its environment through non-specific mechanisms of tolerance, regarding to non-specific anti stress enzymes involved with degradation, as GST, and changes in structure of lipid membrane, perhaps preventing the entrance of the herbicide in the cell in its toxic configuration. *E. coli* DH5-α, already a model for different studies in bacterial metabolism and adaptation, can also be used for the study of other enzymatic and structural systems related to herbicides tolerance and adaptation in contaminated environments, through phenotypic plasticity of those systems.

## References

[1] DayanFE, CantrellCL, DukeSO (2009) Natural products in crop protection. Bioorg Med Chem 17: 4022–4034.1921608010.1016/j.bmc.2009.01.046

[2] ArmasEDD, MonteiroRTR, AntunesPM, SantosMAPFD, CamargoPBD, et al (2007) Diagnóstico espaço-temporal da ocorrência de herbicidas nas águas superficiais e sedimentos do Rio Corumbataí e principais afluentes. Quím Nova 30: 1119–1127.

[3] SandsDC, MorrisCE, DratzEA, PilgeramA (2009) Elevating optimal human nutrition to a central goal of plant breeding and production of plant-based foods. Plant Sci 117: 377–389.10.1016/j.plantsci.2009.07.011PMC286613720467463

[4] Kiely T, Donaldson D, Grube A (2004) Pesticides industry sales and usage: 2000 and 2001 market estimate. US Environmental Protection Agency 1–33.

[5] JiangL, HuangJ, LiangL, ZhengPY, YangH (2008) Mobility of prometryne in soil as affected by dissolved organic matter. J Agric Food Chem 56: 11933–11940.1905337810.1021/jf8023134

[6] Lopez-PerezGC, Arias-EstevezM, Lopez-PeriagoE, Soto-GonzalezB, Cancho-GrandeB, et al (2006) Dynamics of pesticides in potato crops. J Agric Food Chem 54: 1797–1803.1650683610.1021/jf0525737

[7] MartinsPF, MartinezCO, CarvalhoG, CarneiroOIB, AzevedoRA, et al (2007) Selection of microorganisms degrading s-metolachlor herbicide. Braz Arch Biol Technol 50: 153–159.

[8] SharmaD, NagpalA, PakadeYB, KatnoriaJK (2010) Analytical methods for estimation of organophosphorus pesticide residues in fruits and vegetables: A review. Talanta 82: 1077–1089.2080130210.1016/j.talanta.2010.06.043

[9] CyconM, MarkowiczA, Piotrowska-SegetZ (2013) Structural and functional diversity of bacterial community in soil treated with the herbicide napropamide estimated by the DGGE, CLPP and r/K-strategy approaches. Appl Soil Ecol 72: 242–250.

[10] HernándezM, JiaZ, ConradR, SeegerM (2011) Simazine application inhibits nitrification and changes the ammonia-oxidizing bacterial communities in a fertilized agricultural soil. FEMS Microbiol Ecol 78: 511–519.2206692910.1111/j.1574-6941.2011.01180.x

[11] BonnetJL, BonnemoyF, DusserM, BohatierJ (2008) Toxicity assessment of the herbicides sulcotrione and mesotrione toward two reference environmental microorganisms: *Tetrahymena pyriformis* and *Vibrio fischeri* . Arch Environ Contam Toxicol 55: 576–583.1832272510.1007/s00244-008-9145-2

[12] SilvaTM, StetsMI, MazzettoAM, AndradeFD, PileggiSAV, et al (2007) Degradation of 2,4-D herbicide by microorganisms isolated from Brazilian contaminated soil. Braz J Microbiol 38: 522–525.

[13] MartinsPF, CarvalhoG, GratãoPL, DouradoMN, PileggiM, et al (2011) Effects of the herbicides acetochlor and metolachlor on antioxidant enzymes in soil bacteria. Process Biochem 46: 1186–1195.

[14] AraújoASF, MonteiroRTR, AbarkeliRB (2003) Effect of glyphosate on the microbial activity of two Brazilian soils. Chemosphere 52: 799–804.1275778010.1016/S0045-6535(03)00266-2

[15] GratãoPL, PolleA, LeaPJ, AzevedoRA (2005) Making the life of heavy metal-stressed plants a little easier. Funct Plant Biol 32: 481–494.10.1071/FP0501632689149

[16] ZhangY, MengD, WangZ, GuoH, WangY, et al (2012) Oxidative stress response in atrazine-degrading bacteria exposed to atrazine. J Haz Mater 229–230: 434–438.10.1016/j.jhazmat.2012.05.05422704773

[17] MonteiroCC, CarvalhoRF, GratãoPL, CarvalhoG, TezottoT, et al (2011) Biochemical responses of the ethylene-insensitive *Never ripe* tomato mutant subjected to cadmium and sodium stresses. Environ Exp Bot 71: 306–320.

[18] CiaMC, GuimarãesACR, MediciLO, ChabregasSM, AzevedoRA (2012) Antioxidant responses to water deficit by drought-tolerant and sensitive sugarcane varieties. Ann Appl Biol 161: 313–324.

[19] AllocatiN, FavaloroB, MasulliM, AlexeyevMF, Di IlioC (2003) Proteus mirabilis glutathione S-transferase B1-1 is involved in protective mechanisms against oxidative and chemical stresses. Biochem J 373: 305–311.1266713910.1042/BJ20030184PMC1223472

[20] GhelfiA, GaziolaSA, CiaMC, ChabregasSM, FalcoMC, et al (2011) Cloning, expression, molecular modelling and docking analysis of glutathione transferase from *Saccharum officinarum* . Ann Appl Biol 159: 267–280.

[21] AllocatiN, FedericiL, MasulliM, Di IlioC (2009) Glutathione transferases in bacteria. Febs J 276: 58–75.1901685210.1111/j.1742-4658.2008.06743.x

[22] MitchellG, BartlettDW, FraserTEM, HawkesTR, HoltDC, et al (2001) Mesotrione: a new selective herbicide for use in maize. Pest Manag Sci 57: 120–128.1145564210.1002/1526-4998(200102)57:2<120::AID-PS254>3.0.CO;2-E

[23] NorrisSR, BarretteT, DellaPennaD (1995) Genetic dissection of carotenoid synthesis in *Arabidopsis* defines plastoquinone as an essential component of phytoene desaturation. Plant Cell 7: 2139–2149.871862410.1105/tpc.7.12.2139PMC161068

[24] BarrettM (1995) Metabolism of herbicides by cytochrome P450 in corn. Drug Metabol Drug Interact 12: 299–315.882085810.1515/dmdi.1995.12.3-4.299

[25] NordbyJN, WilliamsMM, PatakyJK, RiechersDE, LutzJD (2008) A common genetic basis in sweet corn inbred Cr1 for cross sensitivity to multiple cytochrome P450-metabolized herbicides. Weed Sci 56: 376–382.

[26] HatziosKK, BurgosN (2004) Metabolism-based herbicide resistance: regulationby safeners. Weed Sci 52: 454–467.

[27] PicketCB (1989) Glutathione S-transferases: gene structure, regulation, and biological function. Annu Rev Biochem 58: 743–764.267302010.1146/annurev.bi.58.070189.003523

[28] OakleyA (2011) Glutathione transferases: a structural perspective. Drug Metab Rev 43: 138–151.2142869710.3109/03602532.2011.558093

[29] GauduP, FontecaveM (1994) The NADPH: sulfite reductase of *Escherichia coli* is a paraquat reductase. Eur J Biochem 226: 459–463.800156310.1111/j.1432-1033.1994.tb20070.x

[30] AlfernessP, WiebeL (2002) Determination of mesotrione residues and metabolites in crops, soil, and water by liquid chromatography with fluorescence detection. J Agric Food Chem 50: 3926–3934.1208386010.1021/jf011696y

[31] DurandS, SancelmeM, Besse-HogganP, CombourieuB (2010) Biodegradation pathway of mesotrione: complementarities of NMR, LC-NMR and LC-MS for qualitative and quantitative metabolic profiling. Chemosphere 81: 372–380.2069268210.1016/j.chemosphere.2010.07.017

[32] PileggiM, PileggiSAV, OlchanheskiLR, SilvaPAG, GonzalezAMM, et al (2012) Isolation of mesotrione-degrading bacteria from aquatic environments in Brazil. Chemosphere 86: 1127–1132.2224506010.1016/j.chemosphere.2011.12.041

[33] CrouzetO, BatissonI, Besse-HogganP, BonnemoyF, BardotC, et al (2010) Response of soil microbial communities to the herbicide mesotrione: a dose-effect microcosm approach. Soil Biol Biochem 42: 193–202.

[34] BotelhoRG, FroesCM, SantosJB (2012) Toxicity of herbicides on *Escherichia coli* growth. Braz J Biol 72: 141–146.2243739410.1590/s1519-69842012000100016

[35] SondiI, SondiBS (2004) Silver nanoparticles as antimicrobial agent: a case study on *E. coli* as a model for Gram-negative bacteria. J Coll Int Sci 275: 177–182.10.1016/j.jcis.2004.02.01215158396

[36] WilliamsJA, CarnesAE, HodgsonCP (2009) Plasmid DNA vaccine vector design: impact on efficacy, safety and upstream production. Biotec Adv 27: 353–370.10.1016/j.biotechadv.2009.02.003PMC269333519233255

[37] HeathRL, PackerL (1968) Photoperoxidation in isolated chloroplasts. I. Kinetics and stoichiometry of fatty acid peroxidation. Arch Biochem Biophys 125: 189–198.565542510.1016/0003-9861(68)90654-1

[38] GarciaJS, GratãoPL, AzevedoRA, ArrudaMAZ (2006) Metal contamination effects on sunflower (*Helianthus annuus L*.) growth and protein expression in leaves during development. J Agric Food Chem 54: 8623–8630.1706184310.1021/jf061593l

[39] BradfordMM (1976) A rapid and sensitive method for the quantification of microgram quantities of protein utilizing the principle of protein-dye binding. Anal Biochem 72: 248–254.94205110.1016/0003-2697(76)90527-3

[40] GratãoPL, MonteiroCC, AntunesAM, PeresLEP, AzevedoRA (2008) Acquired tolerance of tomato (*Lycopersicon esculentum* cv. Micro-Tom) plants to cadmium-induced stress. Ann Appl Biol 153: 321–333.

[41] BeauchampC, FridovichI (1971) Superoxide Dismutase: improved assays and an assay applicable to acrylamide gels. Anal Biochem 287: 276–287.10.1016/0003-2697(71)90370-84943714

[42] MediciLO, AzevedoRA, SmithRJ, LeaPJ (2004) The influence of nitrogen supply on antioxidant enzymes in plant roots. Funct Plant Biol 31: 1–9.10.1071/FP0313032688875

[43] KrausTE, MckersieBD, FletcherRA (1995) Paclobutrazol-induced tolerance of wheat leaves to paraquat may involve increased antioxidant enzyme activity. J Plant Physiol 145: 570–576.

[44] ZablotowiczRM, HoaglandRE, LockeMA, HickeyWJ (1995) Glutathione-s-transferase activity and metabolism of glutathione conjugates by rhizosphere bacteria. Appl Environ Microbiol 61: 1054–1060.1653495610.1128/aem.61.3.1054-1060.1995PMC1388388

[45] BlighEG, DyerWJ (1959) A rapid method of total lipid extraction and purification. Can J Biochem Phys 37: 911–917.10.1139/o59-09913671378

[46] SouzaML, WackettLWP, MillsKL, MandelbaumRT, SadowskyMJ (1995) Cloning, characterization, and expression of a gene region from *Pseudomonas* sp. Strain ADP involved in the dechlorination of atrazine. Appl Environ Microbiol 61: 3373–3378.757464610.1128/aem.61.9.3373-3378.1995PMC167616

[47] PennaTCV, IshiiM, SouzaLC, CholewaO (2004) Expression of green fluorescent protein (GFPuv) in *Escherichia coli* DH5-α, under different growth Conditions. African J Biotec 3: 105–111.

[48] GreenbergJT, ManachP, ChouJ, JosephyD, DempleB (1990) Positive control of a global antioxidant defense regulon activated by superoxide-generating agents in *Escherichia coli* . Proc Natl Acad Sci USA 87: 6181–6185.169671810.1073/pnas.87.16.6181PMC54496

[49] Isarankura-Na-AyudhyaP, Isarankura-Na-AyudhyaC, YainoyS, ThippakornC, SinghagamolW, et al (2010) Proteomic alterations of *Escherichia coli* by paraquat. EXCLI J 9: 108–118.29255394PMC5698890

[50] LizukaM, InoueY, MurataK, KimuraA (1989) Purification and some properties of glutathione S-transferase from *Escherichia coli* B. J Bacteriol. 171: 6039–6042.10.1128/jb.171.11.6039-6042.1989PMC2104692553668

[51] BatissonI, CrouzetO, Besse-HogganP, SancelmeM, MangotJF, et al (2009) Isolation and characterization of mesotrione-degrading *Bacillus* sp. from soil. Environ Poll 157: 1195–1201.10.1016/j.envpol.2008.12.00919121884

[52] DurandS, AmatoP, SancelmeM, DelortAM, CombourieuB, et al (2006) First isolation and characterization of a bacterial strain that biotransforms the herbicide mesotrione. Lett Appl Microbiol 43: 222–228.1686990910.1111/j.1472-765X.2006.01923.x

[53] BalaguéC, SturtzN, DuffardR, DuffardAME (2001) Effect of 2,4- dichlorophenoxyacetic acid herbicide on *Escherichia coli* growth, chemical composition and cellular envelope. Environ Toxicol 16: 43–53.1134554410.1002/1522-7278(2001)16:1<43::aid-tox50>3.0.co;2-r

[54] LimaES, AbdallaDSP (2001) Peroxidação lipídica: mecanismos e avaliação em amostras biológicas. Braz J Pharm Sci 37: 293–303.

[55] BögerP, MatthesB, SchmalfubJ (2000) Towards the primary target of chloroacetamides - new findings pave the way. Pest Manag Sci 56: 497–508.

[56] SánchezM, GarbiC, Martínez-ÁlvarezR, OrtizLT, AllendeJL, et al (2005) Klebsiella planticola strain DSZ mineralizes simazine: physiological adaptations involved in the process. Appl Microbiol Biotechnol 66: 589–596.1552619610.1007/s00253-004-1735-y

[57] AzevedoRA, AlasRM, SmithRJ, LeaPJ (1998) Response of antioxidant enzymes to transfer from elevated carbon dioxide to air and ozone fumigation, in the leaves and roots of wild-type and a catalase-deficient mutant of barley. Physiol Plant 104: 280–292.

[58] JungIL, KimIG (2003) Transcription of ahpC, katG, and katE genes in *Escherichia coli* is regulated by polyamines: polyamine-deficient mutant sensitive to H_2_O_2_-induced oxidative damage. Biochem Biophys Res Commun 301: 915–922.1258979910.1016/s0006-291x(03)00064-0

[59] NagyI, CompernolleF, GhysK, VanderleydenJ, DemotJ (1995) A single cytochrome P-450 system is involved in degradation of the herbicides EPTC (*s*-ethyl dipropylthiocarbamate) and atrazine by *Rhodococcus* sp. strain NI86/21. Appl Environ Microbiol 61: 2056–2060.764604910.1128/aem.61.5.2056-2060.1995PMC167476

[60] ShaoZQ, BehkiR (1995) Cloning of the genes for degradation of the herbicides EPTC (*s*-ethyl dipropylthiocarbamate) and atrazine from *Rhodococcus* sp. strain TE1. Appl Environ Microbiol 61: 2061–2065.764605010.1128/aem.61.5.2061-2065.1995PMC167477

[61] Fournier J, Soulas G, Parekh N (1997) Main microbial mechanisms of pesticide degradation in soils. In: Tarradellas J (ed) Soil ecotoxicology. Lewis Publishers CRC, New York, pp 85–116.

[62] BusJS, GibsonJE (1984) Paraquat: model for oxidant-initiated toxicity. Environ Health Perspect 55: 37–46.632967410.1289/ehp.845537PMC1568364

[63] MaXX, JiangYL, HeYX, BaoR, ChenY, et al (2009) Structures of yeast glutathione-S-transferase Gtt2 reveal a new catalytic type of GST family. EMBO Reps 10: 1320–1326.10.1038/embor.2009.216PMC279920419851333

[64] SkopelitouK, DhavalaP, PapageorgiouAC, LabrouNE (2012) A glutathione transferase from *Agrobacterium tumefaciens* reveals a novel class of bacterial GST superfamily. PloS One 7: e34263.2249678510.1371/journal.pone.0034263PMC3319563

[65] Van EerdLL, HaoglandRE, HallJC (2003) Pesticide metabolism in plants and microorganisms. Weed Sci 51: 472–495.

[66] McGuinnessMC, MazurkiewiczV, BrennanE, DowlingDN (2007) Dechlorination of pesticide by a specific bacterial glutathione S-transferase. Eng Life Sci 7: 611–615.

[67] CumminsI, AndonNL, HaynesPA, ParkM, FisherWH, et al (2011) Multiple roles for plant glutathione transferases in xenobiotic detoxification. Drug Metab Rev 43: 266–280.2142593910.3109/03602532.2011.552910

